The article "Staged Nursing Intervention: The Effect of the Compliance in Liver Cancer Patients with Interventional Therapy" was retracted in 2023. Reasons: signs of a paper mill; suspected computer-generated content; unreliable results or conclusions; concerns about the data.

# Staged Nursing Intervention: The Effect of the Compliance in Liver Cancer Patients with Interventional Therapy

**DOI:** 10.1155/2022/7517821

**Published:** 2022-03-28

**Authors:** Limin Zhang, Xinsheng Li

**Affiliations:** Department of Hepatobiliary Surgery, the Fourth Hospital Affiliated to Hebei Medical University, Shijiazhuang, Hebei Province, China

## Abstract

**Objective:**

To evaluate the effect of the compliance in liver cancer patients with interventional therapy in the use of staged nursing intervention.

**Methods:**

A total of sixty liver cancer patients with interventional therapy were enrolled from January 2019 to December 2020. All patients were randomized to the control group (*n* = 30) and the experimental group (*n* = 30); routine nursing intervention and staged nursing intervention were conducted, respectively. The characteristics of compliance, psychological state, and other related indicators were recorded and compared.

**Results:**

The experimental group experienced lower VAS scores and higher treatment compliance. After intervention, both groups observed obvious reductions in the self-rating anxiety scale (SAS) scores, self-rating depression scale (SDS), and Pittsburgh Sleep Quality Index (PSQI) scores, while those were markedly lower in the experimental group (all *P* < 0.05). The experimental group yielded a significantly lower complication rate than the control group (*P* < 0.05).

**Conclusion:**

In liver cancer patients with interventional therapy, staged nursing intervention could effectively relieve the pain, reduce the incidence of complications, and timely eliminate the negative emotion, thus playing a vital impact on the prognosis, worthy of further promotion.

## 1. Introduction

Liver cancer is a common malignant tumor in the clinic with both high morbidity and mortality, which has a considerable impact on the safety and quality of life. Currently, the most common first-line treatment strategy is the use of interventional therapy, which could inject the anticancer drugs or embolization agents into the hepatic artery through femoral artery intubation, assisted by angiography, digital subtraction, and other imaging devices, thereby conducting a minimally invasive approach to the local lesions [1]. Recent developments in interventional therapy have highlighted the merits that it could repeat many times, effectively relieve the symptoms, and prolong the survival period [2–5]; however, the actual therapeutic effect largely depends on the treatment compliance [6]. In addition, previous research has revealed the poor clinical treatment effect associated with negative emotions. Diversity nursing and comfort nursing are often used in clinical rehabilitation nursing, but they lack accuracy and standardization, which affect the rehabilitation effect to a certain extent [7, 8]. The comprehensive and systematic nursing intervention has received considerable attention in improving psychological state and treatment compliance. Given that, we would deeply explore the application of staged nursing intervention in liver cancer patients with interventional therapy, thus providing a theoretical reference for improving the clinical treatment compliance. We carried out phased nursing according to the operation stage, and the results were reported as follows.

## 2. Materials and Methodology

### 2.1. General Information

We enrolled 60 liver cancer patients with interventional therapy in our hospital from January 2019 to December 2020. The computer generates 60 random numbers and then carries out random number sorting. Nos. 1–30 is the control group and Nos. 31–60 is the experimental group. Make a random number card and seal it in an opaque envelope. The patients entered the study after signing the informed consent, opened the envelope according to their entry order, and were randomly assigned to two groups, with 30 cases in each group. The ethics committee of our hospital had approved the study. There was no between-group difference in the general data of the two groups, which was comparable (*P* > 0.05). as given in Table 1.

### 2.2. Inclusion Criteria

The inclusion criteria were as follows: conformed to the diagnosis of live cancer with CT, ultrasound, and pathological examination, received interventional therapy for the first time, and patients and their families had signed written informed consent.

### 2.3. Exclusion Criteria

The exclusion criteria were as follows: with the surgical history of liver cancer treatment, complicated with ascites, jaundice, and other serious complications, with liver dysfunction such as cirrhosis, unable to cooperate or refused to cooperate with the investigator, estimated survival <3 months, and pregnant or lactating.

### 2.4. Methods

The control group received routine nursing intervention as follows: assisted patients to complete various examinations and carry out routine postoperative nursing, introduces the purpose, methods, and precautions of interventional surgery to patients, eliminates doubts, negativity, and pessimism, and enhances the confidence to overcome the disease. Second, guide the patients to lie flat for 24 hours after operation, extend the limbs on the puncture side, recover the limb activities after 24 hours, and fast for 4 hours before operation. Introduce the relevant knowledge of liver cancer and the identification of complications to their families and patients, so as to find out the changes of the disease in time. Take medicine according to the doctor's advice and avoid taking drugs that damage the liver.

The experimental group received staged nursing intervention as follows.

1. Psychiatric nursing: most patients were filled with panic, anxiety, and pessimism when established the diagnosis of liver cancer. So, the nursing staff should comprehensively assess the patient's psychological state and implement the following measures. First, timely communicated with patients to inform them of the treatment experience and successful cases. Second, established a friendly relationship with patients and their families. Third, created a relaxed, cheerful, and warm ward environment as possible. Fourth, gave more encouragement, support, and comfort to patients. Fifth, encouraged family members to give patients more emotional support and comfort, thus improving cooperation degree.
2. Nursing intervention before intervention therapy: first, matched the daily diet reasonably, chose digestible liquid food or semiliquid food for the patients, and reminded the patients to fast 4 hours before surgery. Second, assisted the patient in completing various preoperative examinations according to the doctor's instructions, including blood routine, ECG, ultrasound, blood pressure, intraoperative limb, puncture site. Third, timely pacified the patient's preoperative tension.
3. Nursing intervention in interventional operation: patients undergoing interventional therapy might suffer from liver dysfunction due to hypoxia, ischemia, or drug effects, which can lead to lethargy or coma. Therefore, the nurse needed to promptly protect the liver treatment, paid attention to observe the patient's blood, urine volume, skin color, and consciousness changes, and reminded the patient to take more rest and stay warm.
4. Nursing intervention after intervention therapy: for hematoma or bleeding at the puncture site, made the patient lie supine with hip joint straightened and pressed with sandbag for 12 hours (bending of the operative limb or lying on the side was strictly prohibited within 12 hours). Then, observed the body temperature and skin color changes, recorded the dorsal foot artery pulse, and prevented the formation of venous thrombosis. Grasped the precursor of gastrointestinal bleeding and turned the head to one side when the patient had nausea and vomiting. After treatment, the patient might have infectious fever due to coagulant necrosis within the tumor. Adopted ice to physically cool the patient, and antibiotics should be given in severe cases. After interventional treatment, patients might have different degrees of physical pain. The nurse needed to correctly evaluate the pain of patients and relieve the pain by distracting the patients. If the patients were unable to bear the pain, appropriate medication could be adopted.

### 2.5. Observed Indicators

The researchers collected the following data at the time of patient enrollment and discharge:

1. Evaluation of the pain: the visual analogue scale (VAS) was conducted to evaluate the pain. A score of 0–3 indicated tolerable mild pain, 4–6 indicated tolerable but the sleep was affected, and 7–10 indicated intolerable intense pain.
2. Evaluation of the treatment compliance: the treatment compliance was evaluated in terms of medication compliance, regular review, reasonable diet, smoking and alcohol abstinence, and self-evaluation. Complete compliance indicated fully implemented, noncompliance indicated fail to carry out more than four items as required, and the rest are partial compliance. Compliance rate = (complete compliance + partial compliance)/total number × 100%.
3. Evaluation of the psychological states: the psychological states were evaluated with the self-rating anxiety scale (SAS) scores, self-rating depression scale (SDS). SAS and SDS are divided into 20 items, respectively, and the four-level scoring method is adopted. The cutoff value of SAS standard score is 53 points. The cutoff value of SDS standard score is 50 points; the higher the score, the worse the emotion.
4. Evaluation of the sleep quality: the sleep quality was evaluated with the Pittsburgh Sleep Quality Index (PSQI) scores with a total score of 21 points. The lower the score, the better the sleep quality.
5. Incidence of complications: the complications, including gastrointestinal bleeding, infection, and hepatic encephalopathy, were recorded, and the total complications incidence was calculated.

### 2.6. Statistical Methods

Continuous data and categorical data were summarized with the use of ($\bar{x}$ ± *s*) and (*n*, (%)). The comparisons were performed with the *t*-test and chi-square test, respectively. We defined *P* value less than 0.05 as a statistical difference. SPSS 21.0 was adopted for the data analysis.

## 3. Results

### 3.1. Comparison of the VAS Scores of the Two Groups

The experimental group experienced lower VAS scores than the control group (*P* < 0.05), as given in Table 2.

### 3.2. Comparison of the Treatment Compliance of the Two Groups

The experimental group obtained higher treatment compliance than the control group (*P* < 0.05), as given in Table 3.

### 3.3. Comparison of the Score of SAS and SDS of the Two Groups

After intervention, both groups observed obvious reductions in the score of SAS and SDS, while the scores were all markedly lower in the experimental group than the control group (all *P* < 0.05), as shown in Figures 1 and 2.

### 3.4. Comparison of the PSQI Scores of the Two Groups

After intervention, both groups observed obvious reductions in the PSQI scores, while the PSQI scores were markedly lower in the experimental group than the control group (all *P* < 0.05), as shown in Figure 3.

### 3.5. Comparison of the Complications of the Two Groups

The experimental group yielded a significantly lower complications rate than the control group (*P* < 0.05), as given in Table 4.

## 4. Discussion

Liver cancer is a malignant tumor that originated from hepatocellular with a long disease course and is difficult to cure. Recent progression in lifestyle, diet structure, and mental stress has led liver cancer occurrence in patients gradually younger and incidence increased year by year. Patients are prone to anxiety, depression, inferiority, and other negative emotions with the establishment of the diagnosis, which will directly affect the treatment outcome and even lead to deterioration. Of particular concern is the stealthiness of liver cancer that most patients are diagnosed in the middle and advanced stages and lost the opportunity of surgical treatment. Previous research findings have verified interventional therapy as the most effective method for liver cancer, with the advantages of wide indication, definite curative effect, and repeatability [9]. However, the long treatment process of liver cancer is a great test for both physical and mental conditions. When faced the liver cancer, it is difficult to change the social role and adjust the psychological gap, which will not only trigger a series of physical stress response but also greatly reduce treatment compliance. The term “compliance” has been used to refer to whether the treatment behavior of the patient is consistent with the treatment guidance of the doctor, mainly involving following the doctor's advice, changing the bad life behavior, and regular review [10–12]. With low compliance, the treatment effect is limited and even life-threatening. Interventional treatment will directly bring severe pain, which is also a strong psychological stress source [13]. Thus, the psychological state plays a vital impact in treatment compliance. Therefore, we introduced the staged nursing intervention focused on the characteristics of different stages of liver cancer treatment and carried out the nursing plan from both the psychological and physical health dimensions, thus improving the overall treatment effect. The academic literature on psychological care has revealed that if individuals lack good psychological support and coping methods in a high emergency state, the degree of psychological damage is twice that of ordinary people. Therefore, nursing should vary from disease to disease, from person to person, and from stage to stage, thus meeting pathological needs in diversified forms.

In this study, staged nursing intervention was carried out for patients in the experimental group, while routine nursing intervention in the control group. The results showed that the experimental group experienced lower VAS scores and higher treatment compliance; after intervention, both groups observed obvious reductions in the SAS scores, SDS scores, and PSQI scores, while those were markedly lower in the experimental group; the experimental group yielded a significantly lower complications rate than the control group. The comprehensive analysis of the above results indicated that phased nursing intervention could significantly improve treatment compliance with verified clinical efficacy. These results were in line with previous research, which conducted staged nursing intervention to enhance psychological endurance, improve treatment confidence, and promote treatment compliance for patients with interventional treatment of liver cancer [14].

Taken together, in liver cancer patients with interventional therapy, staged nursing intervention could effectively relieve the pain, reduce the incidence of complications, and timely eliminate the negative emotion, thus playing a vital impact on the prognosis, which is worthy of further promotion.

## Figures and Tables

**Figure 1:** Comparison of the VAS scores of the two groups. The horizontal axis is before the intervention and three months after the intervention, and the vertical axis is the scores. The VAS scores of the control group before intervention and 3 months after intervention are (54.3 ± 8.5) and (48.7 ± 3.1), respectively. Those of the experimental group are (54.1 ± 8.4) and (35.6 ± 2.8), respectively. ^∗^Significant difference comparing 3 months after intervention treatment with before treatment (*t* = 3.390 and 11.32; *P*=0.0013 and <0.001). ^∗∗^Significant difference comparing the experimental group with the control group (*t* = 17.18, *P* < 0.001).

**Figure 2:** Comparison of the SDS scores of the two groups. The horizontal axis is before the intervention and three months after the intervention, and the vertical axis is the scores. The SDS scores of the control group before intervention and 3 months after intervention are (59.9 ± 7.5) and (48.5 ± 3.6), respectively. Those of the experimental group are (60.1 ± 7.7) and (35.6 ± 2.8), respectively. ^*∗*^Significant difference comparing 3 months after intervention treatment with before treatment (*t* = 7.506 and 16.36; all *P* < 0.001). ^*∗∗*^Significant difference comparing the experimental group with the control group (*t* = 15.49, *P* < 0.001).

**Figure 3:** Comparison of PSQI scores of the two groups. The horizontal axis is before the intervention and three months after the intervention, and the vertical axis is the scores. The PSQI scores of the control group before intervention and 3 months after intervention are (18.7 ± 2.6) and (10.6 ± 1.5), respectively. Those of the experimental group are (18.3 ± 2.4) and (7.1 ± 1.2), respectively. ^*∗*^Significant difference comparing 3 months after intervention treatment with before treatment (*t* = 14.78 and 22.86; all *P* < 0.001). ^*∗∗*^Significant difference comparing the experimental group with the control group (*t* = 9.980, *P* < 0.001).

**Table 1:** The general data of the two groups.

	Control group (*n* = 30)	Experimental group (*n* = 30)	*χ* ^2^/*t*	*P*
Gender (male/female)	19/11	18/12	0.0705	0.791
Age ($\bar{x}$ ± *s*, year)	48.3 ± 4.5	49.1 ± 4.6	0.4637	0.499
Duration ($\bar{x}$ ± *s*, month)	3.3 ± 0.4	3.2 ± 0.6	0.5769	0.451
Tumor size ($\bar{x}$ ± *s*, cm)	4.6 ± 1.2	4.7 ± 1.1	0.1132	0.738
Smoke (yes/no)	12/18	13/17	0.0686	0.793
Drink (yes/no)	21/9	19/11	0.3000	0.584
Resident (country/town)	25/5	23/7	0.4167	0.519

**Table 2:** Comparison of the VAS scores of the two groups (*n*, (%)).

	0–3	4–6	7–10	Tolerable pain
Control group (*n* = 30)	6 (20.00)	7 (23.33)	17 (56.67)	13 (43.33)
Experimental group (*n* = 30)	12 (40.00)	9 (30.00)	9 (30.00)	21 (70.00)
*χ* ^2^				4.3439
*P*				0.037

**Table 3:** Comparison of the treatment compliance of the two groups (*n*, (%)).

	Noncompliance	Partial compliance	Complete compliance	Compliance rate
Control group (*n* = 30)	7 (23.33)	12 (40.00)	11 (36.67)	23 (76.67)
Experimental group (*n* = 30)	1 (3.33)	11 (36.67)	18 (60.00)	29 (96.67)
*χ* ^2^				5.1923
*P*				0.023

**Table 4:** Comparison of the complications of the two groups (*n*, (%)).

	Gastrointestinal bleeding	Infection	Hepatic encephalopathy	Total incidence
Control group (*n* = 37)	4 (13.33)	3 (10.00)	2 (6.67)	9 (30.00)
Intervention group (*n* = 37)	2 (6.67)	0 (0)	0 (0)	2 (6.67)
*χ* ^2^				5.4545
*P*				0.020

## Data Availability

The datasets used to support this study are available from the corresponding author upon request.
